# Smart Health Monitoring and Management System for Organizations Using Radio-Frequency Identification (RFID) Technology in Hospitals or Emergency Applications

**DOI:** 10.1155/2022/2177548

**Published:** 2022-08-01

**Authors:** Yaw-Wen Kuo, Yung-Chung Tsao, Web-Chang Chien, Yuh-Ming Huang, Lun-De Liao

**Affiliations:** ^1^Department of Electrical Engineering, National Chi Nan University, Nantou, Taiwan; ^2^Institute of Biomedical Engineering and Nanomedicine, National Health Research Institutes, Zhunan, Taiwan; ^3^Computer & Network Center, National Chi Nan University, Nantou, Taiwan; ^4^Department of Computer Science and Information Engineering, National Chi Nan University, Nantou, Taiwan

## Abstract

In the public health domain, healthcare systems are a crucial part of the economy, transportation, education, health infrastructure, and military of any country. In this study, a system is proposed to implement smart people management, monitoring, and tracking processes that can be used in hospitals to automate and organize information management. For disease management in a public setting, measuring forehead temperatures is a standard method of identifying people for further treatment. To prevent disease transmission on campuses or in any public space, daily temperature checks for everyone have been mandated at the entrances to many public spaces. Although this task can be performed in seconds for an individual, substantial human resources are required to perform temperature checks for all people arriving at one or more specified checkpoints each day during an epidemic. As a result, a smart measuring, monitoring, and management system is urgently needed. We propose a complete solution that includes current Internet of Things technology that can be used in hospitals or any public space to automate and organize information management operations. This system offers a cost-effective means of enhancing reliability, privacy, and security for healthcare record management. One attractive feature of the system is its low cost due to the use of off-the-shelf devices and sensors that can be sourced and operated in our region. Recorded measurements of vital sig/ns are presented via a compact, user-friendly interface that can be monitored remotely. Because the proposed solution is based on mature existing hardware modules and software packages, any experienced information technology professional can quickly build an analogous monitoring and management system by following the instructions presented in this paper.

## 1. Introduction

In the public health domain, healthcare systems are a crucial part of the economy, transportation, education, health infrastructure, and military of a country. Recently, healthcare system researchers have been searching for new tools to serve people's needs in a reliable, secure, and cost-effective manner. In addition to wearing face masks, frequent handwashing with soap and water, and using hand sanitizer as preventative measures for disease management in a public setting, temperature measurement is a simple and effective health monitoring method for identifying people for further treatment. We consider the situation in Taiwan as an example. Since February 2020, due to the emergence of COVID-19, the national policy has been to measure the temperatures of employees and students every day during the pandemic. This task is time-consuming, as are the associated data collection and recording tasks. The scenario at universities is especially complicated. In academic settings ranging from kindergartens to senior high schools, students simultaneously pass through only one or two entrance points each day. Therefore, all temperature checks can be conducted during a single period of time in the morning. However, a university campus is an open space where students arrive at different buildings and entrances at different times, which makes the temperature measurement process extremely difficult to manage. The related measurement tasks generally require the reallocation of manpower or the hiring of short-term workers. Moreover, this task exposes the people who perform it to a risky environment. Thus, automated temperature measurement is necessary to reduce the manpower requirements for epidemic mitigation.

Data management is another related issue. Management needs to know the number of students or employees who have had their temperatures measured, and it needs to develop ways to control admission into buildings or classrooms. We consider a simple scenario in which a person undergoes a temperature check in building A. When this person goes to another building, this task does not need to be repeated, and only a simple screener is needed outside the entrance. The temperature measurement is recorded by a backend information system that interacts with screeners and manages data.

If the outbreak of an epidemic exceeds the world's expectations, eventually, all countries may face the same challenges with regard to containing the outbreak through an all out effort. In addition to national policies and actions, any self-management method employed by a society or organization can aid in burden relief. Fortunately, existing Internet of Things (IoT) technologies [1–10] and measurement techniques [11–18] provide abundant resources and design ideas for constructing a quick solution based on existing modules, equipment, and software packages. In addition, automation systems can also be found in the literature [19–25] for body temperature measurement. However, the feasibility is questionable because the authors integrated some types of temperature sensors without evaluation accuracy. Moreover, user privacy and integration with the existing information system are not addressed. This paper proposes a system based on hardware components that are easy to purchase commercially. With a certified forehead thermometer adopted, we do not need to compensate for raw data and conduct complex evaluation processes. Additionally, the selected open-source software packages can be accessed via the Internet.

Figure 1 illustrates the proposed system architecture, which consists of two types of hardware devices and a software gateway. An autothermometer can automatically measure an arriving person's forehead temperature after their radio-frequency identification (RFID) card is detected. After applying the optical character recognition (OCR) process to a photograph of the result displayed on the thermometer screen, the device uploads the unique ID (UID) of the RFID card and the recognized temperature value to the software gateway via the Message Queuing Telemetry Transport (MQTT) protocol [11]. The software gateway stores the incoming message in the database and interacts with the organization's private information system, which maintains the mappings between the UIDs and personal data (the mechanism that records the temperature value attached to the corresponding personal record falls outside the scope of this study). A card screener, which can be deployed at the entrance of a building, for example, is also activated when an RFID card is detected. The screener retrieves the status currently associated with the detected UID by querying the software gateway via the MQTT protocol. The retrieved status is displayed on the liquid-crystal display (LCD), and a beeping sound is triggered. In addition to supporting entrance control, the data that are collected by the screener can be used to trace a confirmed case during the incubation period. In summary, the proposed system serves as a subsystem of the broader campus information system that interacts with the physical world. A new temperature record higher than 37.5°C triggers an immediate notification to the school nurse, who will then take responsibility for any necessary follow-up procedures. The administrators can perform further data analysis by accessing a web user interface page of the private campus system.

The major contribution of this paper is the proposal of a quick and reliable solution for building a health monitoring and management system based on forehead temperature measurements. Users take measurements with well-designed self-service autothermometers, which also act as a bridge to the backend information system. Automatic data delivery achieves the goal of immediate notification and easy analysis. The rest of this paper is organized as follows: Section 2 describes the construction of the two hardware devices.  Section 3 presents the programs that run on the two devices and the software gateway.  Section 4 demonstrates our prototyping efforts and reports the experimental results. Conclusions are presented in Section 5.

## 2. Methods

### 2.1. Autothermometer

Initially, we planned to use an infrared (IR) thermometer from Melexis [12, 19] to measure body temperature; this approach is similar to the method employed in many other projects shown on YouTube. However, after assembling the necessary modules, we discovered that employing an IR thermometer sensor alone is not as easy as we initially thought. Intensive testing showed that the output value depended not only on the skin temperature but also on the ambient temperature, measurement location, and distance to the measured surface. We could not identify an easy way to adjust the readings to ensure consistent output, as achieved by commercial forehead thermometers. Thus, an alternative plan was implemented using an existing forehead thermometer.

The final version of the autothermometer consists of seven components: a forehead thermometer, a Raspberry Pi device, a camera module, an RFID reader, a servo motor, a buzzer, and an ultrasonic distance sensor, as shown in Figure 2. Any forehead thermometer will suffice, but its mounting should be adjusted accordingly. A Raspberry Pi 3B controller, a common Linux-based embedded system platform with many general-purpose I/O (GPIO) pins, is utilized in this device. With proper software packages installed, the device can process images acquired by the attached camera. Typically, all members of a large organization such as a university use badges or student cards for personal identification. RFID tags are often embedded in these badges or cards and are used to record a person's time of entry into a building or to gain admission to restricted areas, such as libraries, gyms, and laboratories. During an epidemic, associating daily temperature data with a UID is a valid approach for health monitoring and management. The RFID reader adopted in this system is an RC522 reader from NXP Semiconductors [13]. After a UID is detected by the RC522 module, the thermometer is triggered when the distance between the thermometer and the user has decreased beyond a certain threshold. A US-100 ultrasonic sensor module is adopted for this purpose. Once the distance is within the threshold, the thermometer is triggered by the servo motor (model MG996R).

The Raspberry Pi device has a dedicated port for a camera module. The complete hardware wiring schematic of the other four components is shown in Figure 3. The middle box in this figure represents the GPIO pin J8 header. The reader is referred to [14] for the detailed definition of each pin. The RC522 RFID module is connected to the serial peripheral interface (SPI) bus, and the ultrasonic sensor, buzzer, and servo motor are controlled with GPIO pins. The servo position is controlled by a pulse-width modulation (PWM) signal. The buzzer generates a sound when the control pin is toggled. The frequency of the generated sound varies with the toggling frequency. Different tones can be used to notify the user about different events. The ultrasonic sensor requires one input pin and one output pin. The sensor, which is triggered by a pulse from the trigger pin with a duration of 10 *µ*s, generates a signal at a frequency of 40 kHz, and the echo pin then outputs a pulse with a duration that is proportional to the distance between the sensor and the user. Let *t* be the pulse duration from the echo pin. The distance can be approximated as follows:

(1) $$\begin{array}{c} \text{distance in cm}=t^{*}\frac{1000000}{58}. \end{array}$$

When the user is sufficiently close to the thermometer, the duty cycle of the PWM signal is slightly changed to generate a physical movement that triggers the thermometer to record the user's temperature. After approximately 0.5 s, the Raspberry Pi device takes a picture of the result displayed on the screen of the thermometer and begins to process the image for number recognition. The recognized temperature value, UID, and media access control (MAC) address of the Raspberry Pi device are then combined to form a JavaScript Object Notation (JSON) [15] string, which is then transmitted via the MQTT protocol.

The current autothermometer design is based on an engineering approach. It is also possible to control a thermometer by directly accessing its internal circuitry; doing so would allow the system to be more compact in size and faster in response time, but the system design would then be specific to a particular thermometer. Considering the variable availability of thermometers, this paper presents an alternative approach to support flexibility in thermometer selection. Thus, the presented design methodology will still be applicable if readers choose to use other handheld thermometers, although the housing and program parameters should be adjusted accordingly.

### 2.2. Card Screener

Currently, more than 20 temperature check stations are in operation at National Chi Nan University, and each station is equipped with a thermometer for temperature measurement and data uploading. If a person passes a temperature check, they are stamped on the back of one hand. If they move to another building, then the inspector at that building only looks at the stamp. The inspector can ask a person without a stamp to have their forehead temperature measured. Although stamping provides a quick way to screen for people who require temperature measurements, the stamp can be too blurry to be identified, and inspectors are exposed to risk because they directly interact with students and personnel.

The card screener is designed to address this scenario. Because the data are stored in a database, a query based on the UID can be issued to retrieve the personal status of any individual. Since screeners must be deployed in many locations, low cost is an important design requirement. Accordingly, the WeMos D1 mini is selected because it is cheap, compact, and mature; it is based on the ESP8266 Wi-Fi module, which has been extensively employed in many IoT sensors deployed by our laboratory. The components of the card screener are illustrated in Figure 4. In addition to the WeMos D1 mini, an RFID reader, a buzzer, and an interintegrated circuit (I2C) LCD are needed. The hardware wiring is shown in Figure 5. The RC522 reader is controlled by the SPI, and the buzzer is toggled by a GPIO pin (D4). The LCD is controlled by the I2C interface.

With the help of the card screener, an inspector can monitor temperatures from a safe distance. In the future, we plan to integrate the card screener into the door control system by means of the unused pin D3. In this way, admission control can be performed automatically without the need to deploy inspectors. Another advantage of utilizing card screeners is that they facilitate the creation of individual footprints. If a confirmed case is identified, management can quickly identify the affected areas by tracking the footprints of the corresponding individual.

## 3. Results

In the system architecture shown in Figure 1, the MQTT broker and database already exist in our current IoT platform. Similar systems could be established based on existing free services, purchased services, or self-built services. An MQTT-based IoT architecture is commonly adopted because the MQTT protocol is less complex than the Hypertext Transfer Protocol (HTTP) [16], which means that less powerful controllers can be employed for remote IoT sensors. Another advantage is that we can decouple the database from the Internet by hosting the database on a private network. Without a public Internet Protocol (IP) address, the database is hidden from anyone on the Internet. This approach can significantly reduce the possibility of network attacks. Accordingly, we need to employ a software gateway for protocol translation and data manipulation.

An MQTT system consists of one broker and several clients. A client can publish messages with specific topics to the broker. A client can also subscribe to particular topics. After the broker receives a message, it forwards the message to every client that is subscribed to a topic that matches the topic field of that message. Three quality-of-service (QoS) levels are supported by MQTT systems. QoS level 0 is the simplest; at this level, the broker does not send an acknowledgment to the sender. In this case, the sender does not know whether a transmission is successful. At QoS level 1, the broker returns a *PUBACK* message to the sender. If the sender does not receive the *PUBACK* message, the original message is resent. If the *PUBACK* message is lost, then the broker will receive a duplicate message due to retransmission. The upper-level software needs to filter out these duplicate messages. QoS level 2 is the most complex approach; at this level, both the sender and the receiver are informed about a successful transmission. After the broker receives a message, it returns a *PUBREC* message. After receiving the *PUBREC* message, the sender can delete the data and sends a *PUBREL* message. After receiving the *PUBREL* message, the broker returns a *PUBCOMP* message. Retransmission occurs if the sender does not receive either the *PUBREC* message or the *PUBCOMP* message. In our scenario, the broker and software gateway are executed on the same virtual machine, and the virtual machine and database are directly connected to a 10 Gbps Ethernet network. We can assume that almost no packet loss occurs during the transmission process shown on the right-hand side of Figure 1. In contrast, the autothermometer and card screener are based on Wi-Fi by default. As will be subsequently addressed, careful treatment is necessary to ensure reliable transmission to and from these devices.

### 3.1. Software Design for the Autothermometer

The Raspberry Pi device is a Linux-based embedded system. The functionality developed in this project is based on Python 3 because many resources for this programming language are available online. The main task is to automatically trigger the forehead thermometer when a user approaches. The main flowchart is illustrated in Figure 6.

The program starts automatically after the system is powered up and runs continuously. After initialization, the program continuously checks whether an RFID card is detected. If a valid UID is received, the device starts measuring the distance to the individual with the ultrasonic module. Once the distance is less than a specified threshold, the program adjusts the PWM signal fed to the control pin of the servo motor. The resulting physical movement triggers the forehead thermometer to obtain one measurement. After approximately 0.5 s, the program takes a picture with the camera and performs OCR on the image after cropping it in accordance with a predefined location. The program returns to the card scanning stage if the OCR result is invalid. If the temperature value is higher than 37.5°C, which means that the user has a fever, then an e-mail notification is sent to the school nurse or manager. The extracted value is delivered to the software gateway via the MQTT protocol in JSON format. This step ends the entire cycle, and the program then returns to the beginning of the main loop.

For RFID reading, the program periodically polls the status of the RC522 Python library. The Python Adafruit hcsr04 library is not recommended for this ultrasonic sensor because it requires high central processing unit (CPU) usage. The operation of the ultrasonic sensor is extremely simple, as previously described, and requires only two GPIO pins. The first GPIO pin acts as an output pin that generates a 10-*µ*s trigger pulse, and the second GPIO pin acts as an input pin to measure the duration of the pulse generated by the module. This task is performed periodically until the calculated distance is below the threshold. The GPIO pin configured as the output is used to generate a PWM signal for the servo motor. The program slightly increases the duty cycle for approximately 0.3 s to trigger the thermometer, and then, the servo motor returns to its normal position after the duty cycle is reset to the initial value.

After approximately 0.5 s, depending on the type of thermometer, the camera acquires one image for the OCR process to extract the result from the thermometer screen. Initially, we chose to use the PyTesseract library, which is based on Google's Tesseract-OCR engine [17], a powerful tool for multilanguage recognition. We utilized the model for a seven-segment display. However, this model can recognize only numerical characters, whereas the thermometer we use also displays letters; for example, it displays “Lo” when the temperature is below 36°C and “Hi” when the temperature exceeds 42°C. The Tesseract-OCR engine converts these two strings into number strings, which can lead to unpredictable results. Therefore, we have newly implemented a straightforward OCR algorithm. Because the region of interest for this device is fixed, our new algorithm attempts to determine each digit by checking for the existence of each display segment.  Figure 7(a) shows the numbering scheme for the segments and the corresponding rectangular areas to be checked. Because the distance between the camera and the thermometer screen is only approximately 10 cm, the captured image will be blurry and noisy. To obtain a clear binary image, we adopt the two-step thresholding method from the Open-Source Computer Vision Library (OpenCV) [18]. The cropped image is first blurred by a Gaussian filter, and then Otsu thresholding [18] is applied. The binarization result is generally satisfactory, as shown on the right-hand side of Figure 7(a). The next step is to determine the symbol for a given digit. If the number of black pixels in a particular rectangle is larger than a certain threshold, the segment that contains that rectangle is considered to exist. Let an integer variable, result, represent the segment detection result. If the *i*th segment exists, then the *i*th bit of *result* is set. Each symbol can thus be represented by a unique value, as shown in Figure 7(b). We employ a Python dictionary to store this mapping relationship. The pseudocode for the process of recognizing a digit is given in Figure 7(c). The program initially checks only the first digit. If an “*L*” or “*H*” is detected, then the checks of the other two digits can be omitted because the output can be determined solely from the first digit. In our application, the LCD brightness can vary considerably. Therefore, we may need to darken the image to obtain a satisfactory result.

We assume that Wi-Fi is utilized by default. Packet loss may cause publishing failure for the MQTT protocol. To mitigate this issue, the program uses QoS level 1 to establish a reliable link to the MQTT broker. The published messages are redirected to the software gateway, which is run on the same virtual machine as the broker. Currently, each MQTT message sent by the autothermometer includes a topic, i.e., *TEMP*, and the following three fields: the Raspberry Pi's MAC address, the user's UID, and the recognized temperature value. The MAC address is used to identify the location of the autothermometer.

### 3.2. Software Design for the Card Screener

As shown in Figure 8, the task of the card screener is relatively simple. The Wi-Fi connection is checked continuously. If the connection is lost, then the device attempts to reconnect to the access point (AP). When a connection exists, the program polls the status of the RC522 module until a valid UID is received. The query task for the status associated with the UID is performed by issuing an MQTT message with the topic *TEMP_CHECK*. Currently, each MQTT message sent by the card screener consists of two fields: the MAC address of the ESP8266 module and the UID. By subscribing to the topic *TEMP_CHECK*, the software gateway can receive these query requests.

The query result is also delivered as an MQTT message issued by the software gateway. In this scenario, the device needs to wait for a response from the software gateway to complete the current round of transmission. We do not use QoS level 2 because of the high protocol overhead that would be incurred. Instead, QoS level 0 is adopted. Although packet loss may occur, robust information delivery can be achieved through retransmission. If no query result is returned within a certain amount of time, then the screener issues another MQTT message. If this process still fails after three attempts, then a warning message is displayed on the LCD screen to notify the user. The user can call the administrator to ask for help. If a query result is returned, then the result is displayed on the LCD screen and may be used to issue a trigger signal to other equipment, such as an automatic door for entrance admission control.

### 3.3. Software Design for the Software Gateway

The backend information system often has an important role in an IoT system for data manipulation. In this project, the software gateway acts as the bridge that connects the hardware devices to the private data services of the university. The software gateway is a Python program that runs on a CentOS-based Linux virtual machine. As illustrated in Figure 9, the software gateway performs two main tasks: processing the MQTT messages generated by the autothermometers and processing the messages from the card screeners.

The software gateway subscribes to the *TEMP* and *TEMP_CHECK* topics when it is executed. An autothermometer sends an MQTT message with the topic *TEMP* after a user forehead temperature is measured, and the message is then forwarded to the software gateway. From a table that contains the mappings between the autothermometer MAC addresses and locations, the software gateway can identify the location of the autothermometer. A record that contains the MAC address, location, UID, and temperature is then stored in the database via a Structured Query Language (SQL) insertion command. All personal and private data are stored in the university computer center. The software gateway can post the record to the private information system of the university using a customized web service application programming interface (API) that was developed by our computer and network center. This record will then be attached to the personal data that correspond to the UID. Regarding message delivery via MQTT, at QoS level 1, the software gateway may receive duplicate messages. Incoming message filtering is therefore required to delete duplicate messages.

The data flow for the card screeners is complex because a message should be returned. As mentioned, QoS level 0 is employed in this case. When a card screener has waited too long for a return message, it publishes the same message again. All screeners use the same topic, *TEMP_CHECK*, and the software gateway is subscribed to it. Because the return message is designated only for the source screener, each screener subscribes to a unique topic constructed using the string “TEMP_CHECK/” followed by its unique MAC address. For each new message, the software gateway also stores this event in the database and queries the status that corresponds to the UID. In addition to the data generated by the autothermometers, personal temperature data may be entered manually via a web page. Therefore, if the query result is empty, then the software gateway needs to query the university information system, which is a task performed by the web service. Currently, each UID has four possible states: (a) invalid, (b) no data for today, (c) OK, and (d) over temperature. The state is transmitted only to the source screener via an MQTT message with the topic “TEMP_CHECK/mac_address.” In this manner, the software gateway can simultaneously serve multiple screeners. After a return message is received, the screener displays the result on the LCD and notifies the user with a corresponding tone.

## 4. Discussion

Although most hardware components and software packages utilized in the presented system are readily available, considerable effort is necessary for performing integration and fine-tuning. For example, the location of the servo motor affects the physical movement of the thermometer. The proper position of the motor can be determined only through repeated experiments. The prototype developed in this research was released after several days of work.  Figure 10 shows an autothermometer assembly with customized wooden housing where the reader can observe how all components were assembled. A real example is shown in Figure 11, which depicts an autothermometer located in the lobby of a student dormitory. Each of the four dormitories is currently equipped with one autothermometer. Students can have their forehead temperatures taken when leaving their dormitory for classes each day. A High-Definition Multimedia Interface (HDMI) screen is attached to the autothermometer to provide a real-time output, and based on this feedback, a user can repeat the measurement process if an invalid value is generated. The most frequently observed error is that the temperature is measured below 36°C, which may occur when a person's hair covers their forehead. The time needed to compute the OCR output can be easily evaluated from the time stamps printed before and after OCR. As shown in Figure 12, approximately 0.7 s is needed to process an image with the Raspberry Pi 3 device. Users reported that they are generally satisfied with the response time because the overall time, including measurement and data uploading, is less than the time needed for the manual temperature check process.

One public health strategy that can be employed during an epidemic period is to measure the forehead temperatures of individuals each day. This precaution can enable people with a fever to immediately seek treatment before transmission can occur. This task is easy to manage for employees but more difficult for students, which is why we designed the card screener. Once additional autothermometers have been deployed, the second stage can begin. At the entrances to restaurants and convenience stores on campus, inspectors can be deployed during busy periods. All individuals must swipe their cards to be granted permission to enter. In addition to displaying the results on a screen, different beep tones are available for notification. These inspectors can thus perform their jobs from a safe distance. As shown in Figure 13, the card screener is relatively simple to assemble. The four possible responses are also depicted at the bottom of Figure 13. The “invalid card” status indicates that the swiped card was not issued by the university. Visitors can use any RFID card to activate any autothermometer, and the measured result will be stored in the database. If the temperature is normal, then the RFID card can be verified by the card screener.

Regarding the durability of this system, the long-term reliability of the system has been evaluated based on the results from multiple stations that have been in operation for a long time. There are currently 11 stations.  Figure 14 shows the daily data counts at each station. During the depicted period, our country required body temperature measurements every day of each week until Friday. In the middle of the month of May, the outbreak level of the epidemic was upgraded to level three, and the mode of instruction changed to online courses. Except for holidays, the system was able to collect more than 1,500 data points on weekdays. The reasons for those failures that occurred during this period were that the motor was broken or the internal forehead thermometer was out of power, though not because of system design issues; therefore, we conclude that this system is reliable. The system durability was evaluated in multisite field deployment. Currently, we have 11 working deployment sites.  Figure 14 plots the daily counts at different sites for six months when taking a temperature measurement each day was a mandatory procedure in our community. The last notable feature of the proposed system is that it enables individuals on campus to be tracked. For example, the activities of one of the authors on April 10 are shown in Figure 15. After we installed four new autothermometers at different stations, a card with UID XXXX1570 was utilized to test their functions. These records were stored in the *TEMP* table. After a few minutes, the same card was scanned by a screener located at the Department of Electrical Engineering. This event was stored in another table named *TEMP_CHECK*. In this manner, user footprints can be generated by querying the *TEMP_CHECK* table for a given UID. If a confirmed case is found, possible candidates for infection can be quickly identified based on this table.

There are two types of failures: false alarms and missed detection. For every measurement higher than 37.5°C, the staff will give the corresponding user a call to clarify his or her actual condition. If there is no concern, the case will be closed. Consequently, a false alarm case is not difficult to manage. On the other hand, a missed detection event is harder to identify. Typically, the root cause is that the user is moving too quickly when the thermometer takes the measurement. This is the main weakness of the proposed system, according to our deployment experience.

## 5. Conclusions

This paper presents a complete system for health monitoring and management. Users can have their temperatures taken by self-service autothermometers that collect data for the system. This approach considerably reduces the manpower requirements for temperature monitoring. Based on this system, management personnel can monitor user health conditions and implement necessary actions, such as real-time care and entrance admission control. The experimental results obtained using our prototype show the ability to successfully collect more than one thousand records each day using 11 deployed autothermometers. The open-source nature of the hardware and all of the software components used in this study makes our system accessible to the community of researchers to build on and improve (https://github.com/ywkuo/Helth-monitoring-and-management-system). In the future, we plan to add the feature of user misbehavior detection to identify whether a user is moving during measurement. Video motion detection is one possible solution for this purpose. We believe that this feature can make the system more reliable.

## Figures and Tables

**Figure 1:** Overall system architecture, including two types of hardware devices and a software gateway.

**Figure 2:** Components of the autothermometer system (from top left): a forehead thermometer, a Raspberry Pi device, a camera module, an RFID reader, a servo motor, a buzzer, and an ultrasonic module.

**Figure 3:** Hardware wiring for the autothermometer.

**Figure 4:** Components of the card screener (from left): a WeMos D1 mini, an RFID reader, a buzzer, and an I2C LCD.

**Figure 5:** Hardware wiring for the card screener.

**Figure 6:** Flowchart of autothermometer operation.

**Figure 7:** Illustration of seven-segment OCR: (a) the definitions of the segment numbers and the seven rectangular areas to be checked, (b) the mapping dictionary for each character, and (c) the pseudocode for digit recognization.

**Figure 8:** Flowchart of card screener operation.

**Figure 9:** Data flow of the autothermometer (a) and card screener (b).

**Figure 10:** Autothermometer assembly.

**Figure 11:** Station set up in the lobby of a student dormitory. The small LCD screen (left part) acts as an interactive user interface.

**Figure 12:** Required computation time for processing an image.

**Figure 13:** Card screener assembly and four possible outputs.

**Figure 14:** Daily counts at different sites for six months.

**Figure 15:** Screenshots of temperature records at different stations (a) and a corresponding footprint record captured by a card screener (b).

## Data Availability

The data used to support the findings of the study can be obtained from the corresponding author upon request.
